The article "A Novel Single Neuron Perceptron with Universal Approximation and XOR Computation Properties" was published in 2014. Journal: Comput Intell Neurosci.

# A Novel Single Neuron Perceptron with Universal Approximation and XOR Computation Properties

**DOI:** 10.1155/2014/746376

**Published:** 2014-04-28

**Authors:** Ehsan Lotfi, M.-R. Akbarzadeh-T

**Affiliations:** ^1^Department of Computer Engineering, Torbat-e-Jam Branch, Islamic Azad University, Torbat-e-Jam, Iran; ^2^Electrical and Computer Engineering Departments, Center of Excellence on Soft Computing and Intelligent Information Processing, Ferdowsi University of Mashhad, Iran

## Abstract

We propose a biologically motivated brain-inspired single neuron perceptron (SNP) with universal approximation and XOR computation properties. This computational model extends the input pattern and is based on the excitatory and inhibitory learning rules inspired from neural connections in the human brain's nervous system. The resulting architecture of SNP can be trained by supervised excitatory and inhibitory online learning rules. The main features of proposed single layer perceptron are universal approximation property and low computational complexity. The method is tested on 6 UCI (University of California, Irvine) pattern recognition and classification datasets. Various comparisons with multilayer perceptron (MLP) with gradient decent backpropagation (GDBP) learning algorithm indicate the superiority of the approach in terms of higher accuracy, lower time, and spatial complexity, as well as faster training. Hence, we believe the proposed approach can be generally applicable to various problems such as in pattern recognition and classification.

## 1. Introduction

In various computer applications such as pattern recognition, classification, and prediction, a learning module can be implemented by various approaches including statistical, structural, and neural approaches. Among these methods, artificial neural networks (ANNs) are inspired by physiological workings of the brain. They are based on mathematical model of single neural cell (neuron) named single neuron perceptron (SNP) and try to resemble the actual networks of neurons in the brain. As computational models, SNP has particular characteristics such as the ability to learn and generalize. Although the multilayer perceptron (MLP) can approximate any functions [1, 2], traditional SNP is not universal approximator. MLP can learn through the error backpropagation algorithm (EBP), whereby the error of output units is propagated back to adjust the connecting weights within the network. In MLP architecture, by increasing the number of neurons in input layer or (and) the number of neurons in output layer or (and) the number of neurons in hidden layer(s), the number of learning parameters and the algorithm computational complexity are significantly increased. This problem is usually referred to as the curse of dimensionality [3, 4]. So many researchers have tried to propose more powerful single layer architectures and faster algorithms such as functional link networks (FLNs) and Levenberg-Marquardt (LM) and its modified and extended versions [5–20].

In contrast to the MLP, SNP and FLNs do not impose high computational complexity and are far from the curse of dimensionality. But because of disregarding the universal approximation property, SNP and FLNs are not very popular in the applications. In contrast to the previse knowledge about SNP, this paper aims to propose a novel SNP model that can solve the XOR problem and we show that it can be universal approximator. Proposed SNP can solve XOR problem only if additional nonlinear operator is used. As illustrated in the next section, the SNP universal approximation property can simply be archived by extending the input patterns and using the nonlinear operator max. Like functional link networks (FLNs) [21], the proposed SNP does not include hidden units or expand the input vector, but guarantees universal approximation. FLNs are single-layer neural networks that can be considered as an alternative approach in the data mining to overcome the complexities associated with MLP [22] but they do not guarantee universal approximation.

The paper is organized as follows. Proposed SNP and universal approximation theorem are proposed in Section 2.  Section 3 presents the numerical results, where the proposed SNP is compared with backpropagation MLP. There are various versions of backpropagation algorithms. In classification problems, we compare with gradient descent backpropagation (GDBP) [23], that is, the standard basic algorithm. Finally, conclusions are made in Section 4.

## 2. Proposed Single Neuron Perceptron

Figure 1 shows the proposed SNP. In the figure, the model is presented as *n* + 1-inputs single-output architecture. The variable *p* is the input pattern and the variable *T* is related target applied in the learning process (3). Let us extend the input pattern as follows:

(1) $$\begin{array}{c} p_{n+1}=\underset{j=1,\ldots ,n}{\max}\left(p_{j}\right). \end{array}$$

Actually, max⁡ operation increases the input dimension to *n* + 1.

So, the new input pattern has *n* + 1 elements. In Figure 1, the input pattern is illustrated by vector *p*_1__≤*j*≤*n*+1_ and the *E*_*o*_ calculated by the following formula is the final output:

(2) $$\begin{array}{c} E_{o}\left(p\right)=f\left(\overset{n+1}{\underset{j=1}{\sum }}w_{j}\times p_{j}+b\right), \end{array}$$

where *f* is activation function and *w*_1_, *w*_2_,…, *w*_*n*+1_, and* b* are adjustable weights. So, error can be achieved as follows:

(3) $$\begin{array}{c} e=T-E_{o} \end{array}$$

and the learning weights can be adjusted by the following excitatory learning rule:

(4) $$\begin{array}{c} w_{j}=w_{j}+\alpha \max\left(e,0\right)p_{j};\;\text{for}\;j=1,\ldots ,n+1 \end{array}$$

and then by the following inhibitory rule:

(5) $$\begin{array}{c} w_{j}=w_{j}-\alpha \max\left(-e,0\right)p_{j};\;\text{for}\;j=1,\ldots ,n+1, \end{array}$$

where *T* is target, *E*_*o*_ is output of network, *e* is related error, and *α* is the learning rate. Also *b* can be trained by

(6) b=b+αmax⁡(e,0),b=b−αmax⁡(−e,0).

It should be added that max operation applied on the input pattern and also in the learning phase has been motivated from computational models of limbic system in the brain [24–26]. Limbic system is an emotional processor in the mammalian brain [27–29]. In these models [24–26], the max operator prepares the output and input of main parts of limbic system.

In summary, the feedforward computation and backward learning algorithm of proposed SNP, in an online form and with* tansig* activation function, is as in Algorithm 1.

In the algorithm, *α* can be picked empirically or changed adaptively during the learning process according to the adaptive learning [30, 31].

The proposed SNP solves the XOR problem. Consider 2−1 architecture with hardlim activation function and by using the following weights: *w*_1_ = −1, *w*_2_ = −2, *v*_3_ = 2, and *b* = −1; thus,

(7) f⌢(1,1)=hardlim(w1×1+w2×1+w3×max⁡(1,1)+b)=0f⌢(0,0)=hardlim(w1×0+w2×0+w3×max⁡(0,0)+b)=0f⌢(1,0)=hardlim(w1×1+w2×0+w3×max⁡(1,0)+b)=1f⌢(0,1)=hardlim(w1×0+w2×1+w3×max⁡⁡(0,1)+b)=1,

where hardlim is calculated by the following formula:

(8) $$\begin{array}{c} \text{hardlim}\left(x\right)=\{\begin{array}{cc} 1 & \text{if}\;\;\left(x\geq 0\right)\\ 0 & \text{otherwise}. \end{array} \end{array}$$

Since $\overset{⌢}{f}$ is in the form of (2), so $\overset{⌢}{f}$ based on SNP can approximate the XOR function. The proposed model has a lower computational complexity than other methods such as spiking neural networks [32] that solved XOR problem. The computational complexity of proposed SNP is *O*(*n*); this is while it profits from very simple questions adjusting the weights.

In the next section, we prove that SNP is a universal approximator and can approximate all real continuous functions.

### 2.1. Universal Approximation Theorem

Let us ignore the activation function from the model and rewrite (2) like this

(9) $$\begin{array}{c} E\left(s\right)=\overset{n}{\underset{j=1}{\sum }}\left(w_{j}\right)\times s_{j}+b. \end{array}$$

Consider *Y* as the set of all equations in form (9) and *d*_*∞*_(*E*_1_, *E*_2_) = sup⁡_*p*∈*U*_⁡|*E*_1_(*p*) − *E*_2_(*p*)| as a submetric; then (*Y*, *d*_*∞*_) is ametric space [33]. The following theorem shows that (*Y*, *d*_*∞*_) is dense in (*C*[*U*], *d*_*∞*_), where *C*[*U*] is the set of all real continues functions defined on *U*.

*SNP Universal Approximation Theorem.* For any given real continuous function *g* on the compact set *U* ⊂ *R* ^*n*^ and arbitrary *ε* > 0, there exists *E* ∈ *Y* such that

(10) $$\begin{array}{c} \underset{p\in U}{\sup}\left|g\left(p\right)-E\left(p\right)\right|<\varepsilon . \end{array}$$

We use the following Stone-Weierstrass theorem to prove the theorem.

*Stone-Weierstrass Theorem (see [33, 34]).* Let *Y* be a set of real continuous functions on compact set *U*. If (1)  *Y* is algebra,that is, the set *Y* is closed under scalar multiplication (the closing under addition and multiplication is not necessary for real continuous functions [34]), (2) *Y* separates points on *U*, that is, for every *x*, *y* ∈ *U* such that *x* ≠ *y*, there exists *E* ∈ *Y* such that *E*(*x*) ≠ *E*(*y*); and (3)  *Z* vanishes at no point of *U*, that is, for each *x* ∈ *U*, there exists *E* ∈ *Y* such that *E*(*x*) ≠ 0, then the uniform closure of *Y* consists of all real continuous functions on *U*; that is, (*Y*, *d*_*∞*_) is dense in (*C*[*U*], *d*_*∞*_). 

*SNP Universal Approximation Proof.* First, we prove that (*Y*, *d*_*∞*_) is algebra. Let *E* ∈ *Y*, for arbitrary *c* ∈ *R*:

(11) E(p)=∑j=1nwjpj+bcE(p)=∑j=1ncwjpj+cb

which is given in form (8). Thus, *cE* ∈ *Y* and (*Y*, *d*_*∞*_) is an algebra.

Next, we prove that (*Y*, *d*_*∞*_) separates the points on* U*. We prove this by constructing a required* E*, for arbitrary *p* ^1^, *p* ^2^ ∈ *U* such that *p* ^1^ ≠ *p* ^2^, and we choose *w*, *v* such that *w*_*j*_ = *p*_*j*_^1^, for  *j* = 1,…, *n* and *v*_*n*+1_ = *w*_*n*+1_ = 0.

Thus,

(12) p1≠p2⟹p1·p1≠p1·p2⟹∑j=1n(wj)pj1≠∑j=1n(wj)pj2⟹E(p1)≠E(p2).

Therefore, (*Y*, *d*_*∞*_) separates the point on *U*.

Finally, we prove that (*Y*, *d*_*∞*_) vanishes at no point of *U*. We choose *w*_*j*_ = 0, for *j* = 1,…, *n*, *v*_*n*+1_ = 0, *w*_*n*+1_ > 0, and *b* = 1.

Since, for all *p* ∈ *R* ^*n*^,

(13) $$\begin{array}{c} \overset{n}{\underset{j=1}{\sum }}\left(w_{j}\right)p_{j}=0 \end{array}$$

and *b* > 0, then, for all *p* ∈ *R* ^*n*^, there exists *E* such that *E*(*p*) ≠ 0.

So, SNP independently from activation function is universal approximator.

## 3. Numerical Results

One parameter that related to computational complexity of a learning method is the number of learning weights in each epoch. The lower number of learning weights concludes lower number of computations and lower computational complexity. To evaluate the number of proposed SNP learning weights with respect to the MLP, we propose a measure named the reducing ratio of number of weights (Rw) as follows:

(14) Rw=(1−Number  Of  Learning  Weights  of  SNP  ModelNumber  Of  Learning  Weights  of  MLP  Model)×100.

The Rw is a measure that can be used to compare the computational complexity of proposed SNP and MPL. The higher Rw shows SNP has a lower number of learning weights. Thus, it has a lower number of computations and so has a lower computational complexity. Additionally, in the classification problems, the accuracy can be a proper performance measure to evaluate the algorithms. This measure is generally expressed as follows:

(15) $$\begin{array}{c} \text{Accuracy}=\frac{\text{Correct}\;\text{Detection}}{\text{All}}. \end{array}$$

For all learning scenarios listed below, the training set contained 70% while the testing set contained 15% of the data and the remaining was used for the validation set. Input patterns have been normalized between [0 1]. Output targets are binary digits (i.e., the single class is labeled by digits “1” and “0,” the two classes are labeled as “01” and “10,” and the three classes are labeled as “001,” “010,” and “100,” and…). Also the initial weights were randomly selected between [0 1].

Here and prior to entering comparative numerical studies, let us analyze the computational complexity. Regarding the proposed learning algorithm, the algorithm adjusts *O*(2*n*) weights for each learning sample, where *n* is number of input attributes. In contrast, computational time is *O*(*cn*) for MLP, where *c* is number of hidden neurons (the lowest *c* is 2). Additionally, GDBP MLP compared here is based on derivative computations which impose high complexity, while the proposed method is derivative free. So, the proposed method has lower computational complexity and higher efficiency with respect to the MLP. This improved computing efficiency can be important for online predictions, especially when the time interval of observations is small.

To test and assess the SNP in classification, 6 single class datasets have been downloaded from UCI (University of California, Irvine) Data Center. In all datasets, the target labeling was binary.  Table 1 shows the information related to the datasets that include the number of attributes and instances. Additionally, the SNP and MLP architectures and the number of learning weights and Rw are presented in the table too. As illustrated in Table 1, SNP reduces the number of learning weights approximately about 50% for each dataset.

In the proposed SNP algorithm, we consider *b* = 0. And the learning parameters values are shown in Table 1. The activation function was* tansig* and the stop criterion in learning process was the maximum epochs, which means the maximum number of epochs has been reached. The maximum and minimum values of each dataset were determined and the scaled data (between 0 and 1) were used to adjust the weights. The training was repeated 10 times and the average of accuracy in test set was recorded.  Figure 2 presents the accuracy average and the confidence interval obtained from SNP and MLP. It is obvious that SNP is more accurate than MLP with GDBP algorithm in some datasets. The results indicated in Figure 2 are based on student's *t*-test with 95% confidence.

Although, according to Figure 2, it seems that GDBP is better in some cases, what is very important in the results is number of learning epochs.  Table 2 shows the learning epoch comparisons. According to Table 2, MLP needs many epochs to reach the results of SNP. It is the main feature of proposed SNP, fast learning with lower computational complexity, that makes it suitable for usage in various applications and especially in online problems.

## 4. Conclusion

In this paper, we prove that a single neuron perceptron (SNP) can solve XOR problem and can be a universal approximator. These features can be achieved by extending input pattern and by using max operator. SNP with this extension ability is a novel computational model of neural cell that is learnt by excitatory and inhibitory rules. This new SNP architecture works with fewer numbers of learning weights. Specifically, it only generates *O*(2*n*) learning weights and only requires *O*(2*n*) operations during each training iteration, where *n* is size of input vector. Furthermore, the universal approximation property is theoretically proved for this architecture. The source code of proposed algorithm is accessible from http://www.bitools.ir/projects.html. In numerical studies, SNP was utilized to classify 6 UCI datasets. The comparisons between proposed SNP and backpropagation MLP present the following conclusions. Firstly, the number of learning parameters of SNP is much lower with respect to the standard MLP. Secondly, in classification problems, the performance of supervised excitatory and inhibitory learning algorithm is higher than gradient descent backpropagation (GDBP). Thirdly, lower computational complexity caused from the fewer learning parameters and faster training of proposed SNP make it suitable for real time classification. In short, SNP is a universal approximator with a simple structure and is motivated by neurophysiological knowledge of the human's brain. We believe, based on the multiple case studies as well as the theoretical results in this report, that SNP can be effectively used in pattern recognition and classification problems.

## Figures and Tables

**Figure 1:** Proposed SNP.

**Figure 2:** Comparisons between SNP and MLP.

**Algorithm 1:** Proposed SNP algorithm.

**Table 1:** Datasets and related learning information.

Dataset		Dataset information			Parameters	ENN model		MLP model		Comparison
ID	Name	Instance	Class	Attribute	Learning rates	Architecture	Weights	Architecture	Weights	Rw
1	Diabetes	768	2	8	0.050	9-1	10	8-2-1	21	52%
2	Heart	270	2	13	0.050	14-1	15	13-2-1	31	51%
3	Pima	768	2	8	0.005	9-1	10	8-2-1	21	52%
4	Ionosphere	351	2	34	0.050	35-1	36	34-2-1	73	50%
5	Sonar	208	2	60	0.0005	61-1	62	60-2-1	125	50%
6	Tic-tac	958	2	9	0.0005	10-1	11	9-2-2	23	52%

**Table 2:** Number of learning epoch comparison.

Model	Proposed SNP	GDBP MLP
Diabetes	6091 ± 1973	9500 ± 1046
Heart	3833 ± 2098	10000 ± 0
Pima	6245 ± 2021	10000 ± 0
Ionosphere	2632 ± 1638	10000 ± 0
Sonar	922 ± 1027	9111 ± 2247
Tic-tac	628 ± 576	9952 ± 98

Average	3392	9760
